# Utilization of HCV Viremic Kidneys with Genotyping/Subtyping-Free Sofosbuvir/Velpatasvir Treatment Strategy: Experience from China

**DOI:** 10.1155/2022/3758744

**Published:** 2022-07-30

**Authors:** Hedong Zhang, Qiuhao Liu, Shanbiao Hu, Mingda Zhong, Fenghua Peng, Yong Guo, Chunhua Fang, Manhua Nie, Liang Tan, Helong Dai, Xubiao Xie, Longkai Peng, Gongbin Lan

**Affiliations:** ^1^Department of Kidney Transplantation, The Second Xiangya Hospital of Central South University, Changsha, Hunan 410011, China; ^2^Clinical Research Center for Organ Transplantation in Hunan Province, Changsha, China; ^3^Clinical Immunology Center, Central South University, Changsha, China

## Abstract

**Background:**

Owing to the advent of pangenotypic direct-acting antiviral agents (DAAs) for hepatitis C virus (HCV) treatment, utilization of HCV-infected deceased donor kidneys with simplified genotyping/subtyping-free sofosbuvir/velpatasvir (SOF/VEL) treatment strategy is now becoming a promising strategy for expanding the organ donor pool.

**Methods:**

This retrospective, comparative, single-center study included HCV viremic donor kidneys that were transplanted to 9 HCV-positive (HCV Ab-positive) recipients (D+/R+ group) and 14 HCV-negative recipients (D+/R- group) from May 2018 to January 2021. Both groups received prophylaxis with SOF/VEL treatment within 1-week posttransplant devoid of HCV genotyping/subtyping. The primary outcomes were sustained virologic response 12 weeks after completion of therapy (SVR12) and graft survival at 1-year posttransplant.

**Results:**

Baseline characteristics were similar between the HCV D+/R- and D+/R+ groups. The mean age of all recipients was 39.09 ± 9.65 (SD) years, and 73.9% were male. A total of 92.9% (13 out of 14) recipients had pretreatment HCV viremia in the D+/R- group. The pretreatment HCV viral load in the D+/R+ group (5.98, log 10 IU/mL; IQR, 5.28-6.53) was significantly higher than that in the D+/R- group (3.61, log 10 IU/mL; IQR, 2.57-4.57). After SOF/VEL treatment, SVR12 was achieved in all recipients, with a 100% 1-year patient and graft survival rates. The D+/R+ group had a higher incidence of abnormal liver function (44.4% vs. 7.1%). No significant difference was observed between the two groups in terms of DGF, acute rejection, ALT, serum creatinine, and eGFR within 1-year posttransplant. No severe adverse events associated with either HCV viremia or SOF/VEL were observed.

**Conclusions:**

Using a simplified genotyping/subtyping-free SOF/VEL treatment strategy, kidneys from hepatitis C viremic donors for both infected and uninfected recipients presented with safe, excellent, and comparable 1-year outcomes, which can safely expand the donor pool. HCV-positive donor kidneys should be utilized regularly, regardless of the recipient's HCV status.

## 1. Introduction

The population of patients with end-stage renal disease (ESRD) is increasing each year in China. The prevalence of dialysis patients increased from 255.11 per million population (PMP) in 2013 to 419.39 PMP in 2017 due to the surge of hypertension and diabetes. The total number of dialysis patients in China was estimated to be over 581,000 in 2017 and is predicted to be over 874,000 by 2025 [1–3]. However, kidney transplantation, which is an optimum renal replacement treatment with lower mortality and improved life quality [4–6], is associated with a severe shortage of transplant organs. In contrast to over 578,000 dialysis patients in 2016 [1], only 9,019 of them were treated with kidney transplantation (7224 deceased donations and 1795 living-related donations) [2].

Due to its large population, China has the largest HCV burden worldwide, with an estimated 8.9 million chronic HCV infections despite the relatively lower HCV incidence compared with the United States [7, 8]. In China, 1b (62.78%) and 2a (17.39%) are the two predominant subtypes, which are also different from US with 1a (51.6%), 1b (26.5%), and 2b (9.8%) [9, 10]. Historically, organs from hepatitis C seropositive donors were associated with unfavorable prognosis posttransplant, including liver failure, kidney dysfunction, coronary vasculopathy, and increased mortality [11–14]. Approximately 500 high-quality kidneys from HCV donors are discarded yearly in the United States [15, 16]. However, recent advances in HCV direct-acting antiviral therapies (DAAs) with over 95% cure rate have made utilization of organs from HCV viremic donors to HCV-negative recipients possible to expand the donor pool [17–22]. The pangenotypic effect of SOF/VEL or GLE/PIB (glecaprevir/pibrentasvir) has provided the possibility of using a simplified genotyping/subtyping-free HCV treatment strategy [23].

Currently in China, HCV viremic donor kidneys still tend to be allocated to HCV-positive recipients or even discarded when no matched HCV-positive recipients are available. HCV NAT (nucleic acid testing)-positive for negative kidney transplantation is scarcely reported among China transplantation centers. With this, this study was aimed at comparing 1-year outcomes in HCV NAT-positive donor kidneys being transplanted to recipients with or without HCV infection in our institution with simplified genotyping/subtyping-free sofosbuvir/velpatasvir (SOF/VEL) treatment strategy to improve the understanding of the feasibility and consequences of allocating HCV NAT-positive donor kidneys to HCV NAT-negative recipients in China.

## 2. Method

### 2.1. Study Design

This retrospective, comparative single-center study included 15 HCV NAT-positive donors, 9 HCV-positive (HCV antibody positive) recipients (D+/R+ group), and 14 HCV-negative recipients (D+/R- group) from May 2018 to January 2021. Seven HCV NAT-positive donor kidneys were allocated to other centers. All data were obtained from the electronic medical record system of our hospital and the China Organ Transplant Response System (COTRS). All deceased donations were obtained after informed consent was signed by their legal guardians. All recipients were informed of the risks and potential expenses associated with HCV viremic donors, agreed on use of clinical data for research purposes, and provided written informed consent. The study was performed in accordance with the Declaration of Helsinki, the principles of Good Clinical Practice, and local regulatory requirements. All study procedures were reviewed and approved by the Ethics Committee of the Second Xiangya Hospital of Central South University.

All recipients were followed up at 1-week interval within 1-month posttransplant; at 2-week interval within 3-month posttransplant; and at 1-month interval within 1-year posttransplant, including physical examination, review of medications, and safety assessments. Routine blood examination, renal function, liver function, urinary sediment test, and drug concentration examination were regularly performed during the follow-up.

The primary outcome was HCV cure at SVR12, which is defined as undetectable HCV RNA at 12-week post-HCV treatment and graft survival at 1-year posttransplant. Secondary outcomes include adverse events of DAA agents, alanine transaminase (ALT) change, renal function, liver function impairment, and patient survival. Liver function impairment is defined as any elevation of ALT/AST/bilirubin. Data on adverse events were extracted from medical records after reviewing the laboratory values and progress notes.

### 2.2. HCV Detection and Treatment

The quantity of HCV RNA in the serum was determined at our hospital laboratory department with a lower limit of quantification at 25 IU/mL. Preemptive 12-week treatment with SOF/VEL started within 1-week posttransplantation for all recipients at their own expense. HCV genotyping/subtyping was not regularly performed and was only planned for patients with SOF/VEL treatment failure. SOF/VEL was selected owing to its pangenotypic effect, less interaction with immunosuppressants, and absence of dose adjustment requirement for patients with renal impairment [23]. Although current data show its safety in patients with severe renal impairment (eGFR < 30 mL/min/1.73 m^2^) and end-stage renal disease on hemodialysis, further safety data are needed since sofosbuvir is mainly eliminated through the renal route [23].

### 2.3. Immunosuppression

All patients received mycophenolate mofetil (MMF; 1 g) and intravenous methylprednisolone (500 mg) before transplantation. Anti-thymocyte globulin or basiliximab was used as induction therapy. Tacrolimus, MMF, and methylprednisolone were administered after the transplantation. The trough concentration of tacrolimus was maintained at 8–10 ng/mL and 7–8 ng/mL during the first 3 months and first year posttransplantation, respectively. MMF was administered at an oral dose of 0.75 g twice a day, and the MMF area under the curve was maintained at 30–60 mg · h/L. Following intravenous methylprednisolone (1.5 g), oral methylprednisolone was administered at an initial dose of 64 mg/day, which was reduced by 8 mg/day and was eventually maintained at 4–8 mg/day.

### 2.4. Statistical Analysis

All statistical analyses were performed using SPSS software, version 22. Continuous variables were presented as means ± standard deviations or as medians with interquartile ranges and were compared using the Mann-Whitney *U* test (for nonnormally distributed variables) or Student's *t*-test. Categorical variables were presented as numbers and percentages and were compared using Fisher's exact test. Statistical significance was set at *P* < 0.05. The glomerular filtration rate was calculated using the Chronic Kidney Disease Epidemiology Collaboration equation.

## 3. Results

Nine HCV NAT-positive to HCV Ab-positive kidney transplants (D+/R+ group) and 14 HCV NAT-positive to HCV Ab-negative kidney transplants (D+/R- group) were performed from May 2018 to January 2021. The baseline characteristics of the donors are described in Table 1. Overall, the donors were well-matched between the two groups in accordance to age, weight, donation type, terminal creatinine, HCV viral load, etc. The mean age of the donors was 47.00 ± 13.67 (SD) years, with a mean weight of 64.22 kg and 82.6% of them were male. The causes of death for all donors were intracerebral hemorrhage (60.9%), head trauma (21.7%), and anoxia (17.4%). The mean donor terminal creatinine and median donor HCV viral load were 107.79 ± 66.58 (SD) *μ*mol/L and 6.37 (log 10 IU/mL; IQR, 5.19-7.35), respectively.

As shown in Table 2, no significant difference was observed between the two groups regarding age, weight, sex, blood type, kidney failure causes, and time of dialysis. The average age of all recipients was 39.09 ± 9.65 (SD) years with a mean weight of 60.41 kg, and 73.9% were men. The major cause of ESRD was glomerulonephritis (82.6%), followed by hypertension (8.7%). The median time of dialysis prior to transplantation was 18 months (IQR, 10-31) months. One recipient in the D+/R- group had a prior transplant. One recipient had a prior diagnosis of HCV and achieved SVR12 with SOF/VEL before kidney transplantation. The mean HLA mismatch for all recipients was 2.44 ± 0.59 (SD). Although the highest pretransplant APRI (AST to platelet ratio index) score in all patients is only 0.57 which shows low risk of significant fibrosis and cirrhosis [24], APRI in D+/R+ group (0.28 ± 0.15) is slightly higher than that in D+/R- group (0.17 ± 0.10) with *P* value at 0.059.

All recipients were given SOF/VEL within 1-week posttransplant and achieved SVR12. Although the HCV infection diagnosis in the D+/R+ group was based on HCV Ab positivity without pretransplant HCV NAT test, the pretreatment HCV viral load in the D+/R+ group (5.98, log 10 IU/mL; IQR, 5.28-6.53) was remarkably higher than that in the D+/R- group (3.61, log 10 IU/mL; IQR, 2.57-4.57) with a *P* value of 0.002. All recipients, except one patient in the D+/R- group, had a positive pretreatment HCV RNA test, which showed a 92.9% (13 out of 14) donor-derived HCV transmission rate in the D+/R- group. The D+/R+ group (44.4%) had a higher incidence of abnormal liver function incidence within 1-year posttransplant than the D+/R- group (7.1%), which might be attributed to prior HCV infection. As shown in Figure 1, ALT level within 1-month posttransplant in the D+/R+ group had a higher degree of variation and tended to converge to a variation similar to the D+/R- group after 1-month posttransplant. No severe adverse events associated with either HCV viremia or SOF/VEL were observed.

All recipients achieved 1-year graft survival and patient survival. There was no statistically significant difference between the two groups in terms of delayed graft function (DGF) incidence, acute rejection incidence, and eGFR at 3- and 6-month posttransplant. Among all recipients, nine (39.1%) patients had DGF, and three (13.0%) experienced acute rejection. As shown in Figure 2, the serum creatinine and eGFR improved in a similar pattern within a year posttransplant between the two groups. This indicated to an unhindered kidney allograft function recovery regardless of recipient HCV status under SOF/VEL therapy.

## 4. Discussion

This single-center retrospective study that utilized HCV viremic donor kidneys resulted in excellent 1-year posttransplantation outcomes regardless of recipient HCV status. All recipients achieved SVR12 with 100% 1-year patient and graft survival with a simplified genotyping/subtyping-free SOF/VEL treatment strategy. Although the D+/R+ group had a higher incidence of abnormal liver function, comparable DGF, acute rejection, ALT, serum creatinine, and eGFR were found between the two groups.

Historically, HCV-infected kidney transplantation recipients are accompanied by inferior allografts and patient outcomes [12, 25]. A study analyzing 33,357 kidney transplantation recipients from 2004 to 2006 in the United States showed that compared with non-HCV infected kidney transplantation recipients, HCV-positive recipients had a higher risk of death (hazard ratio (HR), 1.50; 95% confidence interval (95% CI), 1.28-1.75) and graft failure (HR, 1.26; 95% CI, 1.08-1.47) [25].

The common practice in the pre-DAA era (first DAA agent sofosbuvir was approved in 2013) is to transplant HCV-positive donor kidneys to recipients with pretransplant HCV infection [26]. However, there is a risk when HCV-positive recipients accept HCV-positive donor kidneys. A preexisting HCV infection cannot elicit full protective immunity against reinfection with heterologous or homologous genotypes [27]. HCV superinfection was also observed when HCV-positive recipients accept a kidney that was infected with a different HCV genotype [28].

Transplantation of HCV-positive donor kidneys to HCV-positive recipients has been widely studied way before DAA agents since it could substantially shorten waitlist time and improve patient survival while being easily accepted by recipients [29–34]. A study in 2004 showed that accepting HCV Ab-positive donor kidneys was associated with improved survival compared with the remaining on dialysis among a recipient group with 51.7% HCV Ab-positive rate [33]. In 2010, Morales et al. [34] reported similar 10-year outcomes between HCV Ab-positive recipients who accepted HCV Ab positive versus negative kidneys in terms of patient survival, graft survival, and liver disease.

Between January 2002 and June 2006 of the pre-DAA era, our center performed kidney transplantation on 19 HCV-positive patients with written risk informed consent, including 6 who received kidneys from anti-HCV-positive donors and 13 from seronegative donors. No significant difference was found between the two groups in terms of patient survival, graft survival, and liver impairment [35].

Transplanting HCV-positive donor kidneys to HCV-negative recipients was much more controversial in the pre-DAA era because the long-term outcome was significantly worse on graft and patient survival as compared with transplanting HCV-negative donor kidneys [36]. However, accepting HCV-positive donor kidneys still has a remarkably higher 5-year patient survival rate in contrast to remaining on dialysis [36].

In the DAA era, despite 100% donor-derived HCV viremic rate among HCV-negative recipients, the original THINKER (Transplanting Hepatitis C kidneys Into Negative KidnEy Recipients) trials have achieved 100% SVR12 (defined as an undetectable HCV RNA at 12 weeks posttreatment) and good allograft function in 20 kidney recipients using 12-week course DAA treatment starting on day 3 posttransplantation [19]. The EXPANDER trial has reported similar results in 10 kidney recipients with a 30% HCV viremic rate using DAA treatment initiated prior to transplantation [21]. Of note, the two aforementioned studies suggest that earlier preemptive initiation of DAA treatment might lower the recipient HCV viremic rate. With SOF/VEL 2-day perioperative prophylaxis protocol starting prior to transplantation, Gupta et al. [37] achieved a 30% (3 out of 10) HCV transmission rate from HCV viremic donor to HCV-negative recipients. It is further reduced to 7.5% (3 out of 40) with a 4-day SOF/VEL prophylaxis [37] and 4% (2 out of 50) with a 7-day SOF/VEL protocol [38] which could substantially reduce expenses. In this study, all 102 kidney recipients achieved SVR12 posttreatment and showed similar transplant outcomes in comparison with contemporary HCV-negative donor kidney recipients during short-term follow-up [37, 38]. The combination of early pretransplant DAA prophylaxis initiation, regular posttransplant HCV NAT test, and full-course DAA therapy for recipients with transmission might be the future strategy for utilizing HCV viremic donor kidneys safely, effectively, and economically.

Considering the risk, our center did not perform HCV-positive donor to HCV-negative recipient kidney transplantation until the arrival of pangenotypic DAA agents SOF/VEL (Epclusa), which was first approved by the U.S. Food and Drug Administration on June 2016 [39] and then approved by the China Drug Administration in May 2018 [40].

In this study, SOF/VEL was chosen owing to its pangenotypic effect, less drug-drug interaction with immunosuppressants, and absence of dose adjustment requirement for patients with renal impairment, which makes our simplified genotyping/subtyping-free treatment strategy possible [23]. However, despite its high HCV cure rate (≥95%) and high barrier to resistance, potential treatment failure with the emergence of complex resistance-associated substitutions exists [41, 42]. A slightly lower cure rate was observed in patients with HCV genotype 3b infection and cirrhosis, which accounted for approximately 0.7% cases in China [43]. Once DAA treatment failure occurs, HCV resistance testing and retreatment with a combination of sofosbuvir/velpatasvir/voxilaprevir are recommended [23].

Our study has several limitations. This was a single-center study with a modest sample size. Based on current evidence, initiation of DAA prior to transplant instead of posttransplant might significantly lower the HCV transmission rate [38] which can also reduce the expenses. Additionally, in our study, sofosbuvir, which is mainly eliminated through the renal route, was given for patients with eGFR < 30 mL/min/1.73 m^2^ without severe adverse events. This is consistent with current studies of SOF usage in patients with severe renal impairment [44–46]. Nevertheless, additional precautions should be taken in such cases since higher rates of anemia, deteriorating renal dysfunction, and serious adverse events associated with SOF-containing therapy among patients with eGFR ≤ 45 mL/min/1.73 m^2^ were also reported [47]. Furthermore, considering the high positive predictive value of SVR12 for SVR24, after SVR12, only ALT was closely monitored with each follow-up, while HCV-NAT testing is not regularly performed at 24 weeks post DAA therapy or at 1-year posttransplant. Finally, only the HCV Ab test, rather than HCV RNA, was regularly performed for all recipients pretransplant in our study which may overestimate the HCV viremic recipient percentage [48].

In conclusion, with a simplified genotyping/subtyping-free SOF/VEL treatment strategy, kidneys from hepatitis C viremic donors to both infected and uninfected recipients have safe, excellent, and comparable 1-year outcomes, which represents a method to safely expand the donor pool. The simplified genotyping/subtyping-free sofosbuvir/velpatasvir (SOF/VEL) treatment strategy is easier to conduct and cost efficient which could be the standard procedure with further improvement. Our current HCV-positive to positive allocating strategy should be reviewed and adjusted to avoid discarding surplus of HCV-positive donor kidneys due to lack of appropriate recipients. HCV-positive donor kidneys should also be utilized regularly, regardless of the recipient's HCV status.

## Figures and Tables

**Figure 1:** Posttransplant ALT tests in HCV D+/R- group and D+/R+ group.

**Figure 2:** Comparison of trends in serum creatinine and eGFR posttransplant between HCV D+/R- group and D+/R+ group.

**Table 1:** Donor demographics.

	All (*n* = 23)	D+/R- (*n* = 14)	D+/R+ (*n* = 9)	*P* value
Age, yr, mean (SD)	44.74 ± 13.78	43.29 ± 14.15	47.00 ± 13.67	0.487
Weight, kg, mean (SD)	62.26 ± 12.13	61.00 ± 13.38	64.22 ± 10.33	0.547
Gender, male, *n* (%)	19 (82.6)	13 (92.9)	6 (66.7)	0.260
Cause of death, *n* (%)				0.498
Intracerebral hemorrhage	14 (60.9)	7 (50.0)	7 (77.8)	
Head trauma	5 (21.7)	4 (28.6)	1 (11.2)	
Anoxia	4 (17.4)	3 (21.4)	1 (11.1)	
CIT, hr, median (IQR)	10 (8-11)	10 (8-10)	10 (8-12)	0.363
WIT, min, median (IQR)	2 (1.42-3)	2 (1.48-3)	2 (1.21-3)	0.948
Donor terminal creatinine, *μ*mol/L, mean (SD)	141.63 ± 130.12	163.38 ± 156.91	107.79 ± 66.58	0.430
Donation after cardiac death, *n* (%)	4 (17.4)	3 (21.4)	1 (11.7)	1.00
Donor viral load (log 10 IU/mL), median (IQR)	5.99 (5.45-6.91)	5.84 (5.46-6.92)	6.37 (5.19-7.35)	0.776
KDPI, %, mean (SD)	76.09 ± 16.14	73.71 ± 15.52	79.78 ± 17.30	0.195
KDRI, mean (SD)	1.35 ± 31.12	1.31 ± 0.25	1.41 ± 0.25	0.195

CIT: cold ischemia time; total time from aortic perfusion to reperfusion of the kidneys. WIT: warm ischemia time; asystole to commencement of aortic perfusion.

**Table 2:** Characteristics and outcomes of recipients.

	All (*n* = 23)	D+/R- (*n* = 14)	D+/R+ (*n* = 9)	*P* value
Age, yr, mean (SD)	39.09 ± 9.65	36.29 ± 9.90	43.44 ± 7.86	0.082
Weight, kg, mean (SD)	60.41 ± 9.64	61.44 ± 10.87	58.81 ± 7.66	0.535
Gender, male, *n* (%)	17 (73.9)	10 (71.4)	7 (77.8)	1.000
Cause of ESRD, *n* (%)				0.815
Glomerulonephritis	19 (82.6)	12 (85.7)	7 (77.8)	
Hypertension	2 (8.7)	1 (7.1)	1 (11.1)	
Polycystic kidney disease	1 (4.3)	1 (7.1)	0	
Diabetes mellitus	1 (4.3)	0	1 (11.1)	
Blood type, *n* (%)				0.360
B	8 (34.8)	5 (35.7)	3 (33.3)	
A	7 (30.4)	3 (21.4)	4 (44.4)	
AB	4 (17.4)	4 (28.6)	0	
O	4 (17.4)	2 (14.3)	2 (22.2)	
Dialysis time, mon, median (IQR)	18 (10-31)	16.5 (8.7-28.7)	18 (10.5-40)	0.654
Prior transplant, yes, *n* (%)	1 (4.3)	1(7.1)	0	1.000
HLA mismatch, mean (SD)	2.44 ± 0.59	2.29 ± 0.61	2.67 ± 0.50	0.183
APRI (pretransplantation)	0.21 ± 0.13	0.17 ± 0.10	0.28 ± 0.15	0.059
Induction immunosuppression (*n*, %)				
Basiliximab	7 (0.30)	3 (21.4)	4 (44.4)	0.242
ATG	14 (0.61)	10 (71.4)	4 (44.4)	0.196
No-use	2 (0.09)	1 (7.1)	1 (11.1)	0.742
SVR12	100%	100%	100%	0.801
HCV viral load at treatment start (log 10 IU/mL), median (IQR)	4.26 (2.90-5.90)	3.61 (2.57-4.57)	5.98 (5.28-6.53)	0.002
Abnormal liver function < 1 year, *n* (%)	5 (21.7)	1 (7.1)	4 (44.4)	0.056
ALT at 3-month posttransplant, mean (SD)	19.70 ± 11.39	19.88 ± 9.55	19.41 ± 14.44	0.298
ALT at 6-month posttransplant, mean (SD)	17.80 ± 14.02	16.08 ± 8.73	20.48 ± 20.09	0.801
Delayed graft function, *n* (%)	9 (39.1)	6 (42.9)	3 (33.3)	1.000
Acute rejection < 1 year, *n* (%)	3 (13.0)	2 (14.3)	1 (11.1)	1.000
eGFR at 3-month posttransplant, mean (SD)	65.58 ± 21.72	67.50 ± 22.46	62.59 ± 21.46	0.746
eGFR at 6-month posttransplant, mean (SD)	73.34 ± 25.27	72.73 ± 26.06	74.31 ± 25.53	0.798
1-year death-censored graft survival	100%	100%	100%	
1-year patient survival	100%	100%	100%	

ESRD: end-stage kidney disease; HLA: human leukocyte antigen; eGFR: estimated glomerular filtration rate; APRI: aspartate aminotransferase-to-platelet ratio index; ATG: anti-human T lymphocyte rabbit immunoglobulin.

## Data Availability

The patients data used to support the findings of this study are restricted by the Ethics Committee of the Second Xiangya Hospital of Central South University in order to protect patient privacy. Data are available from Dr. Gongbin Lan (langongbin@csu.edu.cn) for researchers who meet the criteria for access to confidential data.
